The article "Clinical Value of Abdominal Ultrasonography in the Diagnosis of Acute Abdomen in Children" was retracted in 2023. Reasons: signs of a paper mill; suspected computer-generated content; unreliable results or conclusions; lack of ethics approval or compliance.

# Clinical Value of Abdominal Ultrasonography in the Diagnosis of Acute Abdomen in Children

**DOI:** 10.1155/2022/2681543

**Published:** 2022-06-23

**Authors:** Xinxin Xu, Jian Ye

**Affiliations:** ^1^Department of Ultrasound, Wuxi Children's Hospital, Wuxi, Jiangsu 214023, China; ^2^Department of Pediatric Intensive Care Medicine, Wuxi Children's Hospital, Wuxi, Jiangsu 214023, China

## Abstract

In order to study the practical application value of abdominal ultrasonography in the diagnosis and treatment of acute abdomen in children, this study uses the method of collecting clinical actual cases and scientific analysis to estimate the clinical diagnostic value of high-frequency ultrasound and low-frequency ultrasound. In order to further clarify its curative effect and treatment advantages, a retrospective analysis of medical records was conducted, and 95 children with acute abdominal pain and suspected appendicitis who were admitted to a hospital from September 2021 to November 2021 were reviewed. ATIL HD15000 color Doppler ultrasound was used for diagnosis. The results are as follows: the sensitivity, specificity, positive predictive value, and negative predictive value of low-frequency probe in the diagnosis of intussusception in children were 83.61%, 73.33%, 92.73%, and 52.38%, respectively. The sensitivity, specificity, positive predictive value, and negative predictive value in the diagnosis of mesenteric lymphadenitis were 80.00%, 81.97%, 52.17%, and 94.34%, respectively. The sensitivity, specificity, positive predictive value, and negative predictive value of high-frequency probe in the diagnosis of intussusception in children were 93.44%, 80.00%, 95.00%, and 75.00%, respectively. The sensitivity, specificity, positive predictive value, and negative predictive value in the diagnosis of mesenteric lymphadenitis were 93.33%, 95.08%, 82.35%, and 98.31%, respectively. Among the children with appendicitis confirmed by operation and pathology, 69 cases were detected by high-frequency ultrasound and 4 cases were missed (including 3 cases of acute simple appendicitis and 1 case of perforated appendicitis). The false negative was 4%, there was no false positive, and the sensitivity, specificity and accuracy were 95%, 100%, and 96%. In the same cases, 28 cases were detected by low-frequency ultrasound, 45 cases were missed, the false negative was 61%, and there was no false positive. The sensitivity, specificity, and accuracy were 39%, 100%, and 53%. The sensitivity, accuracy, and false negative of high-frequency ultrasound in the diagnosis of acute appendicitis were significantly higher than that of low-frequency ultrasound. This study shows that ultrasound has high accuracy, sensitivity, and specificity in the diagnosis of acute appendicitis. Low-frequency ultrasound can show the whole picture of the disease and the situation in the abdominal cavity, which can better guide the clinical treatment. Color Doppler hemodynamics is a useful supplement to two-dimensional ultrasound, and ultrasound also plays a positive role in the differential diagnosis of acute appendicitis in children.

## 1. Introduction

Pediatric acute abdomen is a common disease in pediatric clinical work. It is the general name of a group of diseases with abdominal pain as the main symptom, as shown in Figure 1. Acute onset and rapid change often endanger the patient's life. Clinically, if we can make correct diagnosis and appropriate treatment in time, we can avoid or reduce complications and serious consequences. However, some of them are difficult to be diagnosed by clinical manifestations alone, and often need imaging assisted diagnosis. X-ray examination and diagnosis of gastrointestinal perforation and intestinal obstruction were reported as early as the 1920s and 1930s. The application was limited due to radioactive hazards. Ultrasound has been used in the diagnosis of acute abdomen in the 1970s, and it has also played a good role in the diagnosis of acute abdomen [1]. With the development of ultrasound technology, especially the application of high-frequency ultrasound in the examination of abdominal diseases, it can clearly show the hierarchical structure of gastrointestinal tract wall. The application of color Doppler ultrasound in the diagnosis of abdominal diseases can display the blood supply of organs and judge whether there is ischemic necrosis. Ultrasound can not only make clear the diagnosis of some acute abdomen through typical ultrasonic manifestations but also be of great value in the differential diagnosis of diseases. Although there are many reports on the application value of ultrasound in adult acute abdomen at home and abroad, its application is limited because it is vulnerable to obesity and abdominal distension [2]. The abdominal wall of children is thin, and the high-frequency probe can clearly show the level of gastrointestinal tract. Combined with the changes of hemodynamics, it is of great significance for clinical diagnosis. This topic systematically summarizes the ultrasonic image characteristics of common pediatric acute abdomen, and studies the advantages of ultrasonic examination.

## 2. Literature Review

Ricci et al. said that acute appendicitis is one of the most common surgical acute abdomen in children. The immune system of children is not yet mature. It progresses rapidly when it is ill and the response to conservative treatment is poor. Therefore, it is very important to make a clear diagnosis in the early stage of the disease and determine the correct timing of surgical intervention [3]. Purcell et al. said that due to the imperfect development of children's nervous system, unclear location of pain, and large dissociation of gastrointestinal tract, the clinical manifestations of acute appendicitis in children vary, which can be similar to almost any kind of acute abdomen or can be covered up by other diseases [4]. Yacine et al. believe that in clinical work, unnecessary surgery is often performed on children due to false positive diagnosis, or diagnosis is omitted due to false negative judgment, resulting in the delay of operation time, perforation, or abscess formation and other adverse conditions that seriously affect the prognosis [5]. However, Jirapinyo and Thompson said that the development of imaging technology has made a qualitative leap in the diagnosis and treatment of many diseases. For acute appendicitis, the traditional routine diagnosis based on clinical history and signs has also gradually changed with the intervention of ultrasound. Ultrasound imaging can make early and rapid etiological diagnosis and differential diagnosis [6]. Eskelinen et al. showed through animal experiments that the ultrasonographic characteristics of the appendix can be displayed by ligating the appendix or appendiceal artery for 30 minutes. Therefore, they believe that ultrasound can be used for the early diagnosis of appendicitis. Ultrasound has high sensitivity (80%–94%), specificity (86%–100%), and accuracy (82%–95%) in the diagnosis of acute appendicitis [7]. Bertozzi et al. believe that ultrasound has the advantages of low price, real-time, and nonradioactivity compared with CT, and is widely used in clinic. After the application of compression method in the diagnosis of appendicitis was officially reported, ultrasonography was used as an auxiliary diagnostic tool, and gradually applied to the diagnosis of various abdominal diseases [8]. Hafiz et al. believe that the emergence of high-frequency ultrasound enables us to have a clearer understanding of abdominal lesions. Recent studies have shown that ultrasound is used to reduce the misoperation rate and complications of appendectomy in children, making ultrasound become the focus of attention and research [9]. Pavlovic et al. believe that ultrasound examination also has shortcomings. For patients with excessive obesity and obvious abdominal flatulence, the compression method is difficult to carry out, so the observation effect of appendix is poor [10]. Yao et al. found that the ultrasonic display rate of acute appendicitis depends on the degree of inflammation. For cellulitis and suppurative appendicitis, the ultrasonic display rate is 100%. When appendicitis is limited to the mucosal layer, the display rate is only 32% [11]. Fei et al. said that ultrasound examination requires high operator experience, especially when the patient has obvious tenderness and cannot stand compression examination, it should distract the patient's attention. In addition, each ultrasound examination generally takes 30 minutes, which is also a major disadvantage [12].

## 3. Research Methods

### 3.1. Use of Instruments

The instrument used is ATIL HDI5000 color Doppler ultrasound diagnostic instrument, and the probe frequencies are 3.5 and 7.5 MHz.

### 3.2. Research Object

From September 2021 to November 2021, 95 patients with acute abdominal pain and suspected appendicitis in a hospital were retrospectively analyzed for their ultrasonography (including two-dimensional ultrasonography, color Doppler, and pulsed Doppler). There were 43 boys and 52 girls, aged 1.5–15 years (average age 4.3 years) [13].

### 3.3. Instruments and Methods

ATIL HDI5000 color Doppler ultrasonic diagnostic instrument is used, and high-frequency linear array probe (frequency 5 ∼ 12Mhz) and low-frequency convex array probe (frequency 3.5 MHz) are configured. Children with acute abdomen do not need to be prepared before examination. Try to keep the children quiet. Take the supine position. First, use the low-frequency convex array probe (frequency 3.5 MHz) to scan the abdominal substantive organs of the children in detail to determine whether there are lesions in each organ. Then, the high-frequency linear array probe (frequency 5 ∼ 12Mhz) was properly pressurized, and the continuous sliding method was performed according to the shape of gastrointestinal tract. The cross section, longitudinal section, and oblique section were scanned to observe the shape, peristalsis, wall thickness, intestinal cavity expansion, mesenteric lymph node abnormal enlargement, free liquid dark area, and abnormal mass in the basin and abdomen. If an abnormal mass is found, the location, size, shape, capsule, internal echo, blood supply, and the relationship with the intestine should be further observed, and the abdominal great vessels should be detected by color Doppler ultrasound. If the value of ultrasonic examination is greatly reduced or there is no positive finding due to too much intestinal gas shielding, a certain disease is highly suspected clinically, and other examination methods such as upper gastrointestinal radiography, CT, and laboratory examination should be carried out. If necessary, ultrasonic reexamination should be carried out after intestinal preparation such as gastric tube exhaust or defecation so as to prevent missed diagnosis.

### 3.4. Ultrasonic Examination Method

Before the examination, ask the medical history in detail and do the abdominal physical examination in person, and do not use sedative drugs. During the examination, children usually take the supine position and sometimes the left lying position in order to find the appendix behind the cecum. First, the abdomen and pelvis were comprehensively scanned with a conventional abdominal probe (3.5 MHz), and then, the suspected lesion area of the child was examined by graded compression with a 7.5 MHz probe [14]. After finding the appendix, observe the shape and size of the appendix, the thickness of the wall, the condition of the open film line, whether there is fecal stone in the cavity, and whether there is tenderness when the probe is pressurized. Measure the length and diameter of the appendix, cross cut the diameter of the appendix (take the front and rear outer walls of the coarsest part of the appendix as the measuring points) and the thickness of the wall. Observe the blood flow distribution at the appendix wall and mesangium with color Doppler, trace the pulse Doppler spectrum, measure vs, VD, and RI, and take the highest blood flow velocity as the recorded value [15]. Continue to explore the right lower abdomen and around the umbilicus with two-dimensional ultrasound to find out whether there are enlarged lymph nodes and free fluid in the abdominal cavity. Pay attention to the lower amplitude, right kidney, gallbladder, portal vein, and pelvic cavity. Girls should pay attention to the situation of uterus, fallopian tube, and ovary. If the appendix is not detected according to the above examination, expand the examination scope to find other reasons [16]. The instrument used in this study is Philips epiq5, the color Doppler ultrasound model, and the frequency of the probe is 5 MHz ∼12Mhz. The children were placed in the supine position. All children first used the low-frequency probe for abdominal scanning and were given longitudinal scanning, transverse scanning, and oblique scanning, focusing on the periumbilical, cecum, right lower abdomen, and pain parts. Then, scan the suspicious key parts with high-frequency probe, conduct multislice scanning, and gradually pressurize scanning. Focus on recording the morphology, internal echo, and aspect ratio of mesenteric lymph nodes, especially for enlarged lymph nodes, check the internal blood flow of lymph nodes, and record the diastolic and systolic blood flow velocity. Observe the abdominal mass and effusion, record the ultrasonic signs such as intussusception, enteritis, intestinal obstruction, and intestinal perforation, highly suspect intussusception in the presence of cannula sign or concentric circle sign, and record the location, size, and mobility of intussusception. At the same time, replace the high-frequency probe, focus on scanning, and record the length and outer diameter of intussusception into the intestine.

### 3.5. Observation Indicators

① The sensitivity, specificity, positive predictive value, and negative predictive value of low-frequency abdominal ultrasound and high-frequency abdominal ultrasound in the diagnosis of acute abdomen in children were compared
② The signs of intussusception and mesenteric lymphadenitis under high-frequency ultrasound were recorded.

### 3.6. Measurement Method of Appendix

A specially assigned person shall measure the long diameter of the isolated appendix (take the blind end and the broken end to measure their straight-line distance, excluding the middle twisted part), the transverse diameter (take the front and rear diameter of the three cross sections at the widest place, and take the average value), and observe the shape, congestion, and swelling degree. Then, cut open, measure the thickness of the wall, and observe whether there is pus, feces, fecal stone, and changes in the membrane layer in the cavity [17]. If it is a perforation type, observe the location of the perforation and the situation in the abdominal cavity.

If it is a periappendiceal abscess, record the size and location of the abscess, and observe the amount and nature of fluid in the cyst.

### 3.7. Postoperative Pathological Records

The postoperative specimens were sent to pathology, and the pathological results were followed up.

### 3.8. Statistical Treatment

SAS was used for statistical analysis. The measurement data were expressed by *t*-test, the data were expressed by mean soil standard deviation, and the counting data were tested by x^2^. All *P* values were one-sided test results, and *P* < 0.05 was considered to have significant difference [18].

## 4. Result Analysis

### 4.1. Ultrasonic Coincidence Rate

Among 136 cases of acute abdomen confirmed by operation, pathology, or clinical treatment, 65 cases of acute mesenteric lymphadenitis, 38 cases of intussusception, 10 cases of acute appendicitis, 10 cases of intestinal malrotation, and 6 cases of intestinal obstruction were diagnosed by ultrasound. The coincidence rate between ultrasound results and pathology or clinical treatment is shown in Table 1.

### 4.2. Diagnostic Accuracy of Low-Frequency Abdominal Ultrasound in Children with Acute Abdomen

The sensitivity, specificity, positive predictive value, and negative predictive value of low-frequency probe in the diagnosis of infantile intussusception were 83.61% (51/61), 73.33% (11/15), 92.73% (51/55), and 52.38% (11/21), respectively. The sensitivity, specificity, positive predictive value, and negative predictive value of mesenteric lymphadenitis were 80.00% (12/15), 81.97% (50/61), 52.17% (12/23), and 94.34% (50/53), respectively (see Table 2).

### 4.3. Diagnostic Accuracy of High-Frequency Abdominal Ultrasound in Children with Acute Abdomen

The sensitivity, specificity, positive predictive value, and negative predictive value of high-frequency probe in the diagnosis of infantile intussusception were 93.44% (57/61), 80.00% (12/15), 95.00% (57/60), and 75.00% (12/16), respectively. The sensitivity, specificity, positive predictive value, and negative predictive value of mesenteric lymphadenitis were 93.33% (14/15), 95.08% (58/61), 82.35% (14/17), and 98.31% (58/59), respectively (see Tables 3 and 4).

### 4.4. Ultrasonic Characteristics of Various Diseases

Among 95 children with clinically suspected appendicitis, 73 cases were acute appendicitis (including 29 cases of simple appendicitis, 21 cases of suppurative appendicitis, 14 cases of gangrenous appendicitis, and 9 cases of peripheral abscess), all of which were confirmed by operation and pathology; 22 children with nonappendicitis (9 cases of mesenteric lymphadenitis, 3 cases of Meckel diverticulitis, 3 cases of acute intussusception, 1 case of ovarian cyst pedicle torsion, 2 cases of small intestinal malignant lymphoma, 2 cases of acute gastroenteritis, and 2 cases of leukemia abdominal hematoma), of which 9 cases were confirmed by operation and pathology, and 13 cases were confirmed by ultrasonography and clinical follow-up [19], as shown in Table 5.

Among 73 children with appendicitis confirmed by operation and pathology, 69 cases were detected by high-frequency ultrasound and 4 cases were missed (including 3 cases of acute simple appendicitis and 1 case of perforated appendicitis). The false negative was 4%, there was no false positive, and the sensitivity, specificity and accuracy were 95%, 100%, and 96%. In the same case, 28 cases were detected by low-frequency ultrasound, 45 cases were missed, the false negative was 61%, and there was no false positive. The sensitivity, specificity, and accuracy were 39%, 100%, and 53%. The sensitivity, accuracy, and false negative of high-frequency ultrasound in the diagnosis of acute appendicitis were significantly higher than that of low-frequency ultrasound. After statistical x^2^ test, the *p* value was <0.05, which was statistically significant [20]. The results are shown in Figure 2.

### 4.5. Changes of Sonogram in Different Development Stages of Acute Appendicitis in Children

The diameter and wall thickness of acute simple and suppurative (including gangrenous) appendicitis were calculated and analyzed by *t*-test. The *P* values were 0.0036 and 0.0020, respectively, both <0.05. The diameter of the appendix was 0.6 cm or 0.5 cm as the dividing point to evaluate simple appendicitis (29 cases). Taking the diameter >0.6 as the boundary point, 21 cases of acute appendicitis were diagnosed and 8 cases were missed. The sensitivity, specificity, and accuracy were 100%, 74%, and 41%, respectively. Taking the diameter >0.5 cm as the boundary point, 27 cases of simple appendicitis were diagnosed and 2 cases were missed. The sensitivity, specificity, and accuracy of diagnosis were 95%, 97%, and 79% [21].

### 4.6. Acute Simple Appendicitis

The appendix is slightly enlarged, with longitudinal section in finger shape and strip shape, cross section in target ring shape, reduced echo of tube wall, slightly thickened linear strong echo in the central hymen and irregular mouth [22]. In 26 cases of acute simple appendicitis, star shaped color blood flow signals were shown on the wall by high-frequency ultrasound data.

### 4.7. Acute Simple Appendicitis

The appendix is obviously enlarged. The vertical section is mostly sausage like and rigid. It is often shown as thickening and expansion of the blind end. The cross section is more obvious target ring or near oval echo area. The internal echo is uneven. The mucosal layer is obviously thickened hyperechoic strip, irregular, tortuous, and interrupted. There are mass fecal stone strong echo, wide liquid dark area, or small dot echo in the cavity, and decreased echo of muscle wall. Short linear or branched abundant blood flow signals can be seen in the appendix wall and surrounding tissues.

### 4.8. Direct Signs

The appendix is thickened and the wall is thickened. The sonogram shows a low echo tubular structure with blind end, with a diameter of ≥ 7 mm, and the wall part is double-layer, with a thickness of ≥ 2 mm. The vertical section image of appendix shape looks like sausage, and the concentric circle can be seen in the cross section. The concentric circle does not disappear when observed under pressure. Appendiceal effusion is characterized by obvious thickening of the appendix, and the lumen is a strip-shaped dark area or low echo area, which is mostly seen in suppurative or gangrenous appendicitis. The dark zone around the appendix is formed by inflammatory exudates accumulated outside the serosa, with a width of 1 ∼ 5 mm and uneven width.

### 4.9. Indirect Signs

Under high-frequency ultrasound, the transverse section of intussusception hypergenesis showed “concentric circle” and the longitudinal section showed “sleeve sign.” More or less mass hyperechoic tissue can be seen around acute suppurative appendicitis, and a small amount of liquid dark area can be seen in or around the appendix. Acute gangrenous appendicitis is surrounded by greater omentum or adhesive intestines. When complicated with perforation, a small or large amount of liquid dark areas can be seen in the intestinal space or lower abdomen near the appendix, with small punctate echoes. Suppurative appendicitis or gangrenous appendicitis is often accompanied by dilation of surrounding intestines and stagnation of contents.

## 5. Conclusion

This study points out that the high-frequency probe can more intuitively display the intestinal situation, overcome the deficiency of false positive detection in low-frequency discussion, and improve more valuable reference opinions for clinical follow-up diagnosis and treatment. The results also showed that the accuracy of high-frequency probe in the diagnosis of intussusception was 90.79% (69/76), which was significantly higher than that of low-frequency probe; Under high-frequency ultrasound, the sign of mesenteric lymphadenitis is enlarged lymph nodes, beaded, and hypoechoic around. By comparing the experimental data, the accuracy of clinical palpation of abdominal lymph nodes is only 58%, and the accuracy of ultrasonic examination of abdominal abnormal lymph nodes can reach 80%–90%, the sensitivity is 60%–70%, and the specificity is more than 90%. The accuracy of ultrasonic measurement of abdominal lymph node diameter can reach 98%. In the results of this study, the accuracy of clinical diagnosis of mesenteric lymphadenitis in children is 69%, and the accuracy of ultrasonography is 100%. It can be seen that the accuracy of diagnosis of mesenteric lymphadenitis is improved due to the intervention of the ultrasound. Finally, this paper believes that the use of high-frequency probe can not only observe the sound image of intussusception but also observe the changes of the internal structure of intussusception and find the position of intussusception. For mesenteric lymphadenitis, the cortical and medullary echo of enlarged lymph nodes can be clearly displayed by high-frequency probe. The diagnostic accuracy of mesenteric lymphadenitis in this study is 94.74% (72/76), and ultrasound also has high accuracy, sensitivity, and specificity in the diagnosis of acute appendicitis. The diameter of appendix is greater than 5 mm and the change of mucosal line is used as clinical evaluation indexes to judge whether early appendicitis was detected by high-frequency ultrasound. In conclusion, high-frequency abdominal ultrasound has high value in the diagnosis of intussusception and mesenteric lymphadenitis in children. Clinically, high-frequency probe examination should be performed after low-frequency large-area abdominal exploration, which can improve the accuracy of clinical diagnosis.

## Figures and Tables

**Figure 1:** Clinical manifestations of acute abdomen in children.

**Figure 2:** Comparison between high-frequency ultrasound and low-frequency ultrasound.

**Table 1:** Diagnostic coincidence rate between ultrasonic results and pathological or clinical results.

Disease species	Pathological or clinical diagnosis	Ultrasonic diagnosis	Compliance rate (%)
Mesenteric lymphadenitis	70	65	92.86
Intussusception	39	38	97.44
Acute appendicitis	11	10	90.91
Intestinal malrotation with midgut torsion	10	10	100
Intestinal obstruction	6	6	100

**Table 2:** Diagnostic accuracy of low-frequency abdominal ultrasound in children with acute abdomen unit: cases.

Low-frequency ultrasound diagnosis		Gold standard		Total
		+	−	
Intussusception	+	51	4	55
	−	10	11	21
	Total	61	15	76
Mesenteric lymphadenitis	+	12	11	23
	−	3	50	53
	Total	15	61	76

**Table 3:** Diagnostic accuracy of high-frequency abdominal ultrasound in children with acute abdomen unit: cases.

High-frequency ultrasound diagnosis		Gold standard		Total
		+	−	
Intussusception	+	57	3	60
	−	4	12	16
	Total	61	15	76
Mesenteric lymphadenitis	+	14	3	17
	−	1	58	59
	Total	15	61	76

**Table 4:** Comparison of diagnostic value of high-frequency and low-frequency abdominal ultrasound in children with acute abdomen.

	Sensitivity	Specificity	Accuracy
*Intussusception in children*			
High-frequency ultrasound	93.44% (57/61)	80.00% (12/15)	90.79% (69/76)
Low-frequency abdomen	83.61% (51/61)	73.33% (11/15)	81.58% (62/76)
*x* ^2^	6.332	4.125	3.554
*P* value	0.001	0.010	0.023

*Mesenteric lymphadenitis*			
High-frequency ultrasound	93.33% (14/15)	95.08% (58/61)	94.74% (72/76)
Low-frequency abdomen	80.00% (12/15)	81.97% (50/61)	81.58% (62/76)
x^2^	5.146	4.265	3.695
*P* value	0	0.011	0.015

**Table 5:** Final diagnosis results.

Final diagnosis result	Number of children
Acute appendicitis	73
Simplification	29
Purulent	21
Gangrenous	14
Peripheral abscess	9
Nonappendicitis lesions	22
Mesenteric lymphadenitis	9
Meckel diverticulitis	3
Acute intussusception	3
Torsion of ovarian cyst pedicle	1
Malignant lymphoma of small intestine	2
Acute gastroenteritis	2
Leukemia abdominal hematoma	2

## Data Availability

The data used to support the findings of this study are available from the corresponding author upon request
